The article "Study on the Conduction Analysis and Blocking Intervention Scheme of Emotional Disorders between Cancer Patients and Their Families" was retracted in 2023. Reasons: unreliable results or conclusions; concerns about the data; concerns about the results or conclusions; concerns about the peer review.

# Study on the Conduction Analysis and Blocking Intervention Scheme of Emotional Disorders between Cancer Patients and Their Families

**DOI:** 10.1155/2022/4820090

**Published:** 2022-04-25

**Authors:** Ling Hu, Xianfeng Zhang, Zizheng Song, Kunjie Wang, Youchao Jia, Jin Song, Lei Su

**Affiliations:** ^1^Department of Medical Oncology, Affiliated Hospital of Hebei University, Hebei Key Laboratory of Cancer Radiotherapy and Chemotherapy, Baoding, Hebei 071000, China; ^2^Department of Nursing, The Sixth People's Hospital of Hebei Province, 572 Dongfeng East Road, Baoding, 071000 Hebei, China; ^3^Department of Radiotherapy, Affiliated Hospital of Hebei University, 212 Yuhua East Road, Baoding071000, Hebei, China

## Abstract

**Objective:**

To analyze the transmission and blocking intervention scheme of emotional disorders between cancer patients and their families.

**Methods:**

About 150 patients with cancer and 150 family members with mood disorders treated in a tertiary hospital in North China from March 2021 to Octobor2021 were enrolled. The patients were randomly assigned into control group and study group. The control group received routine intervention, and the study group received the diagnosis, intervention, and treatment strategies of doctor-patient-affective disorder. The factors related to the transmission of emotional disorders between cancer patients and their families were analyzed, and the alterations of anxiety, depression, social support, and satisfaction of the two groups were compared under different blocking intervention schemes.

**Results:**

(1) Univariate analysis indicated that there were significant differences in family age, family income, sex, location of tumor, course of disease, TNM stage, somatic symptoms, and the incidence of anxiety and depression. There exhibited no significant difference between the gender of the family, the years of education of the family, the occupational status of the family, the relationship between the family and the patient, the mode of payment of the patient's medical expenses, the age of the patient, the mode of treatment of the patient, the degree of knowledge of the disease, and the incidence of anxiety and depression (*P* > 0.05). The anxiety and depression status of relatives were taken as dependent variables, and the age of family members, family income status, sex of patients, location of tumor, course of disease, TNM stage, and physical symptoms of patients were taken as independent variables, and the data were analyzed by Logistic regression analysis. Logistic regression analysis indicated that family income, tumor location, disease course, TNM stage, and somatic symptoms were the risk factors of anxiety and depression in relatives. (2) Comparison of social support status and intergroup, the objective support, subjective support, support utilization, and total score of social support in the study group were higher compared to the control group. In terms of the depression score before intervention, there exhibited no significant difference (*P* > 0.05), but after intervention, the depression score of the two groups decreased, and the depression score of the study group was lower compared to the control group before intervention, 1 week, 2 weeks, 3 weeks, and 4 weeks after intervention (*P* < 0.05). In terms of the anxiety score before intervention, there exhibited no significant difference (*P* > 0.05), but after intervention, the anxiety score of the two groups decreased, and the anxiety score of the study group was lower compared to the control group before intervention, 1 week, 2 weeks, 3 weeks, and 4 weeks after intervention (*P* < 0.05). Comparison of the satisfaction between the two groups and the study group was very satisfied in 56 cases, satisfactory in 14 cases, and general in 5 cases, and the satisfaction rate was 100.00%. The control group was very satisfied in 35 cases, satisfactory in 23 cases, general in 12 cases, and dissatisfied in 5 cases, and the satisfaction rate was 93.33%. The satisfaction of the study group was higher compared to the control group (*P* < 0.05).

The article "Study on the Conduction Analysis and Blocking Intervention Scheme of Emotional Disorders between Cancer Patients and Their Families" was retracted in 2023. Reasons: unreliable results or conclusions; concerns about the data; concerns about the results or conclusions; concerns about the peer review.

**Conclusion:**

Family income, tumor location, course of disease, TNM stage, and somatic symptoms are the risk factors of anxiety and depression in relatives. After establishing the diagnosis, intervention and treatment strategies of doctor-patient-affective disorder, the emotional disorder of family members of cancer patients, is significantly promoted, and the intervention satisfaction is high, so the scheme is worth promoting.

## 1. Introduction

Cancer is a major public health problem that seriously threatens the health of the Chinese population. The annual medical cost caused by cancer is more than 220 billion [1]. Early intervention of patients with negative mood disorders in families with cancer is helpful to promote the prognosis and life quality of cancer patients [2]. The study found that the social concern of emotional disorders of cancer patients and their families is incomplete, lack of multidimensional longitudinal evaluation, establish the integration of hospital, community follow-up and Internet follow-up mechanism, determine the target population, and analyze the influencing factors in real time [3]. Achieve individual transmission analysis, specify blocking intervention measures. Families of cancer patients spend a lot of time and financial expenses in the treatment of negative affective disorders, making it difficult to sustain them in the long term [4]. The establishment of the social assistance system can give full play to the advantages of low-cost and sustainable development [5]. Multiple research data indicate that most caregivers of cancer patients suffer from negative mood disorders during nursing [6]. After integrating and analyzing 192 literatures about the problems of caregivers of cancer patients, some scholars found that the problems faced by caregivers have something in common, such as negative emotion of caregivers, physical health problems, lack of information needs, and lack of social support system [7]. In the study, some scholars reported the care burden of caregivers of advanced cancer patients and summarized the caregiver problems into the following categories, namely, economic problems, psychological burden, and lack of access to information [8]. Some data indicate that cancer caregivers' primary concern in the care process is to alleviate the patient's suffering and deliberately ignore their own problems, preventing most of the negative emotional barriers from being addressed in a timely manner [9]. In a study of 200 family caregivers, scholars found that less than half of the caregivers were willing to seek professional help on their own problems. Therefore, as a professional helper, social workers should provide services for cancer caregivers to help them out of their predicament [10].

The article "Study on the Conduction Analysis and Blocking Intervention Scheme of Emotional Disorders between Cancer Patients and Their Families" was retracted in 2023. Reasons: unreliable results or conclusions; concerns about the data; concerns about the results or conclusions; concerns about the peer review.

The Fifth Plenary session of the 19th CPC Central Committee examined and adopted the “proposal of the CPC Central Committee on the formulation of the 14th five-year Plan for National Economic and Social Development and the long-term goals for 2035” [11] and put forward the notion to “comprehensively promote the construction of a healthy China: further implement the healthy China action, promote the national health promotion policy, provide all-round full-cycle health services for the people, and facilitate health education and chronic disease management.” According to the International Agency for Research on Cancer (IARC), there are about 19.29 million new cancer cases in 2020. There were 4.57 million new cancer cases in China in 2020 [12]. The 2018 National Comprehensive Cancer Network Cancer Pain Management Guide points out that anxiety and depression seriously affect the ability of cancer patients to cope with disease and aggravate cancer progress [13]. The treatment strategies for emotional disorders of cancer patients are drug therapy and psychotherapy, but it is difficult to adhere to it for a long time, and lack of social free relief measures. Cancer also affects the psychological status of family members to varying degrees. In the diagnosis and treatment of cancer, the family members of cancer patients have a low sense of participation and existence, and have serious anxiety, hoping to give companionship and support to the patients when they experience pain [14]. The degree of anxiety and depression of the family members of some cancer patients is higher compared to the patients. The psychological state of family members directly affects the psychology of patients and outcome. Supportive family environment can enhance the disease resistance of cancer patients and reduce the role of stress response [15].

The article "Study on the Conduction Analysis and Blocking Intervention Scheme of Emotional Disorders between Cancer Patients and Their Families" was retracted in 2023. Reasons: unreliable results or conclusions; concerns about the data; concerns about the results or conclusions; concerns about the peer review.

Some scholars early pay attention to the group of cancer patient caregivers, the research content is extensive, and the research results are rich [16]. In the face of difficulties, cancer patients and their relatives are more willing to seek the support of outside forces, such as the government, social institutions, or psychological counsellors, and the vast majority of cancer patients receive help from relevant nursing institutions or hospice care institutions [17]. Therefore, the relationship between patients and caregivers is mostly employment relationship, and less relatives directly undertake the nursing task. Due to different national conditions, the roles of caregivers of cancer patients in China are mostly assumed by relatives, which is quite different from that of other countries [18]. Chinese researches on caregivers of cancer patients are mostly focused on the fields of medicine, nursing, and psychology, and most of the existing researches are theoretical studies, such as caregiver problem diagnosis, demand analysis, and influencing factor analysis, the interventions for the problems are also put forward in the form of suggestions, and most of them are remedial measures based on the caregiver problem. There are relatively few studies on practical intervention for the practical problems of caregivers [19]. Based on this, this study is of great significance to promote the emotional disorders of cancer patients and their families and is of practical value to the cultivation of practical ability of clinical medical students who participate in the intervention treatment program.

## 2. Patients and Methods

### 2.1. General Information

About 150 patients with cancer and 150 family members with mood disorders treated in a tertiary hospital in North China from March 2021 to October 2021 were enrolled. The patients were randomly assigned into the control group and the study group. The control group received routine intervention (*N* = 75), and the research group received the construction of doctor-patient-affective disorder diagnosis, intervention, and treatment mechanism (*N* = 75). In the control group, the age of the patients was 43-74 years old, the average age was 65.53 ± 3.31 years old, the age of the family members of the patients was 35-80 years old, and the average age was 57.48 ± 2.21 years old, containing 32 males and 43 females; in the study group, the age was 44-76 years old, the average age was 65.55 ± 3.44 years old, the family members of the patients aged 35-80 years old, and the average age was 57.31 ± 2.44 years old, containing 31 males and 44 females. There exhibited no statistical significance in the general data of the two groups. This study was permitted by the Medical Ethics Association of our hospital, and all patients noticed informed consent.

The article "Study on the Conduction Analysis and Blocking Intervention Scheme of Emotional Disorders between Cancer Patients and Their Families" was retracted in 2023. Reasons: unreliable results or conclusions; concerns about the data; concerns about the results or conclusions; concerns about the peer review.

The inclusion criteria of cancer patients and their families are as follows: (1) cancer patients and their spouses or children who are mainly responsible for care; (2) cancer patients ≤ 80 years old and their family members ≤ 60 years old; (3) no cognitive impairment and be able to communicate with others; and (4) primary school education or above, can cooperate to complete the research.

Exclusion criteria for cancer patients and their families were as follows: (1) patients with mental illness or patients with other mental disorders, such as mania and schizophrenia; (2) patients with a history of serious heart disease and lung disease; (3) those who have participated in psychological intervention training in the past; (4) those with dysosmia complicated with respiratory diseases, such as asthma and rhinitis; and (5) in the past month, there have been major psychological trauma events, such as bereavement, divorce, and economic problems, which may affect the emotional state of the patients.

### 2.2. Treatment Methods

#### 2.2.1. Survey Tool

Survey tools and analysis methods, self-rating depression scale (CES-D), self-rating anxiety scale (SAS), social support rating scale (SSRS), general situation questionnaire, and patient disease information questionnaire made by the author on the basis of consulting related literature, were used in this survey.

#### 2.2.2. Blocking Intervention Scheme

The control group received routine intervention in the department, issued disease guidance manuals to patients on the day of admission, evaluated admission, patiently carried out health education for patients, and explained to patients matters needing attention in disease-related self-management. Individualized nursing guidance is given, and education is mainly carried out through health education.

On the basis of the control group, the subjects were classified according to the attribution of patients and genera, and the inducing factors of negative emotional disorders were analyzed: (1) on the basis of general health education and guidance, psychological intervention was carried out according to the therapeutic communication system; (2) to set up a psychological intervention team, the members are composed of oncologists, nurses, psychological counselors, and medical student volunteers; (3) to establish a consultation-visit relationship, a good consultation-visit relationship is the basis of the whole work, and the methods of use include emotional experience, identity, and empathy; (4) home intervention is to focus on improving the relationship among family members, establishing a harmonious family, contacting We-chat twice a week, or talking to the patients' family members in the community. Patients are required to communicate with their families for 30 minutes a day, and psychological counselors communicate with patients and their families on the multimedia platform at least once a month; (5) group counseling; (6) to establish a We-chat platform to educate the tumor-related knowledge and promote the patients' family members' awareness of the tumor; and (7) the experimental study lasted for 12 months.

The article "Study on the Conduction Analysis and Blocking Intervention Scheme of Emotional Disorders between Cancer Patients and Their Families" was retracted in 2023. Reasons: unreliable results or conclusions; concerns about the data; concerns about the results or conclusions; concerns about the peer review.

### 2.3. Observation Index

#### 2.3.1. Flow Invocation CES-D

Compiled by Fan Rongping et al. of the National Institute of Mental Health in 1977 [18], the scale is widely employed in epidemiological investigation to screen out subjects with depressive symptoms. Compared with other CES-Ds, it focuses more on individual emotional experience and less on somatic symptoms during depression. CES-D is assessed according to the frequency of corresponding situations or feelings in the past week and consists of 20 questions, containing four reverse questions. The answers are assigned into four levels: (1) none or almost none (no more than one day when such a situation occurs); (2) few (within 1-2 days); (3) often (3-4 days); and (4) almost all the time (5-7 days), score 0, 1, 2, and 3 points, respectively, according to the above order, and reverse mark 3, 2, 1, and 0 points. The scores of 20 questions add up to a total score. In the cooperation group of some areas in China, 1150 people were studied by using CES-D as a norm, the mean value was 11.52. ≥16 points were marked as having depressive symptoms.

#### 2.3.2. SAS

Compiled by Zung in 1971, it was employed to evaluate the subjective feelings of anxiety patients. There were 20 questions, containing 4 reverse scores [19]. The answers were assigned into 4 grades, and the positive scores were 1, 2, 3, and 4, respectively. The reverse score was 4, 3, 2, and 1. The total score of 20 topics was added up to get the total rough score. In the scale cooperation group, 1158 Chinese normal subjects were studied. The results indicated that the average gross score was 29.78 ± 10.07, and the normal upper limit of the total gross score was 40 points.

The article "Study on the Conduction Analysis and Blocking Intervention Scheme of Emotional Disorders between Cancer Patients and Their Families" was retracted in 2023. Reasons: unreliable results or conclusions; concerns about the data; concerns about the results or conclusions; concerns about the peer review.

#### 2.3.3. SSRS

Compiled by Xiao Shuiyuan in 1986 and tested by a large sample of people in the community, it is proved to have good reliability and validity, and it is widely employed in the field of psychosomatic medicine in China [20]. The scale includes three dimensions: objective support (3 items), subjective support (4 items), and utilization of social support (3 items). There are 10 items in the scale, only one item is enrolled for each item of item 1-4 and item 8-10, and items 1, 2, 3, and 4 are enrolled for 1, 2, 3, and 4, respectively, and item 5 is assigned into A, B, C, D, and E5, each item is scored 0-4 from nonsupport to full support. In articles 6 and 7, if you answer “there is no source,” the score will be 0. For those who answer “the following sources,” several sources will be counted. The total score is the sum of 10 items, and the total score ranges from 12 to 66. The higher the score, the higher the social support, lower than 33 points as low social support, 33 to 45 points as average social support, and higher than 45 points as high social support.

#### 2.3.4. General Situation Questionnaire

It includes the gender, age, education level, occupational status, kinship with the patient, family income status, the payment method of patient's medical expenses, patient's sex, age, cancer location, course of disease, cancer stage, the main mode of treatment, and the patient's knowledge of the disease.

### 2.4. Statistical Analysis

The double entry method inputs the survey results into the Epidata3.02 database. SPSS21.0 statistical software was employed to analyze the data. Variance analysis was employed to compare the measurement data between groups, *χ*^2^ test was employed to compare the counting data rate, and multiple linear stepwise regression analysis was employed to screen the factors affecting depression score (*P* < 0.05).

## 3. Results

### 3.1. Factors Affecting the Incidence of Anxiety and Depression in Relatives

There were significant differences in age of family members, family income status, sex of patients, location of tumor, disease course, TNM stage, somatic symptoms, and incidence of anxiety and depression. There exhibited no significant difference between the gender of the family, the years of education of the family, the occupational status of the family, the relationship between the family and the patient, the mode of payment of patient's medical expenses, the age of the patient, the mode of treatment of the patient, the degree of knowledge of the disease, and the incidence of anxiety and depression (*P* > 0.05). All the data results are indicated in Table 1.

The article "Study on the Conduction Analysis and Blocking Intervention Scheme of Emotional Disorders between Cancer Patients and Their Families" was retracted in 2023. Reasons: unreliable results or conclusions; concerns about the data; concerns about the results or conclusions; concerns about the peer review.

### 3.2. Logistic Regression Analysis of Influencing Factors of Anxiety and Depression in Relatives

The anxiety and depression status of relatives were taken as dependent variables, and the age of family members, family income status, sex of patients, location of tumor, course of disease, TNM stage, and physical symptoms of patients were taken as independent variables, and the data were analyzed by Logistic regression analysis. Logistic regression analysis indicated that family income, tumor location, disease course, TNM stage, and somatic symptoms were the risk factors of anxiety and depression in relatives. All the data results are indicated in Table 2.

### 3.3. Comparison of Social Support

The comparison of social support status and intergroup comparison indicated that the objective support, subjective support, support utilization degree, and total score of social support in the study group were higher compared to the control group (*P* < 0.05). All data results are indicated in Table 3.

### 3.4. Depression Score Comparison

Compared with the depression score before intervention, there exhibited no significant difference (*P* > 0.05). After intervention, however, the depression score of the two groups decreased, and the depression score of the study group was lower compared to the control group before intervention, 1 week, 2 weeks, 3 weeks, and 4 weeks after intervention (*P* < 0.05). All the data results are indicated in Table 4.

### 3.5. Comparison of Anxiety Score

Compared with the anxiety score before intervention, there exhibited no significant difference (*P* > 0.05), but after intervention, the anxiety score of the two groups decreased, and the anxiety score of the study group was lower compared to the control group before intervention, 1 week, 2 weeks, 3 weeks, and 4 weeks after intervention, and the difference exhibited statistically significant (*P* < 0.05). The results of all the data are indicated in Table 5.

### 3.6. Comparison of Satisfaction Degree

In the comparison of satisfaction, the study group was very satisfied in 56 cases, satisfactory in 14 cases, and general in 5 cases, and the satisfaction rate was 100.00%. The control group was very satisfied in 35 cases, satisfactory in 23 cases, general in 12 cases, and dissatisfied in 5 cases, and the satisfaction rate was 93.33%. The satisfaction of the study group was higher compared to the control group (*P* < 0.05). All the data results are indicated in Figure 1.

## 4. Discussion

The latest report released by the IARC shows that the number of people suffering from cancer in the world is growing rapidly, with 18.1 million new cancer cases in 2018 [21]. Cancer is on its way to becoming the leading cause of death and illness in the world. The incidence rate of cancer in China is close to the global average level, and the mortality rate is even higher [22]. About 3.929 million people across the country suffered from cancer in 2015, an increase of 125000 over 2014, according to the latest national cancer statistics report released by the National Cancer Center in 2019. In China, an average of more than 10,000 people are diagnosed with cancer every day, and 7.5 people are diagnosed every minute [23]. Through the analysis of previous data, we can see that the incidence and mortality of cancer in China are increasing year by year. In recent years, with the development of science and technology and the improvement of medical quality, the survival time of cancer patients has been prolonged. The World Health Organization (WHO) has classified cancer as a chronic disease. The latest data indicate that the five-year survival rate of malignant tumors in China has increased from 30.9% in 2009 to 40.5% in 2019 [24]. In the past 10 years, the five-year survival rate of cancer patients in China has increased by nearly 10%. As the biggest “obstacle” hindering the extension of life expectancy of Chinese residents, cancer not only causes great physical and mental pain to cancer patients but also a great negative stress event for caregivers of cancer patients. The prolongation of survival time of cancer patients increases the nursing burden of caregivers of cancer patients to some extent, and the pressure of caregivers of cancer patients becomes more heavier [25].

The article "Study on the Conduction Analysis and Blocking Intervention Scheme of Emotional Disorders between Cancer Patients and Their Families" was retracted in 2023. Reasons: unreliable results or conclusions; concerns about the data; concerns about the results or conclusions; concerns about the peer review.

As a stressor, cancer poses a great threat to the physical and mental health of caregivers of cancer patients [26]. Multiple research data indicate that the mental health status of caregivers of cancer patients is not optimistic, and the incidence of mental illness of caregivers of some cancer patients is equal to or even higher compared to cancer patients themselves. Yan Lairong, Wei Hongyan, and Zhang Gong clearly pointed out in the “investigation of mental health status of family members of cancer patients and analysis of related factors” that the family members of cancer patients have psychological disorders to a certain extent. Among them, the score of anxiety level was higher compared to the domestic norm, there was obvious anxiety, and the anxiety degree of some relatives reached the clinical level [27]. However, due to the personal limitations of cancer escorts, some are unable to identify and relieve their anxiety in a timely manner. Over time, this can have an extremely detrimental effect on cancer patient chaperones [28]. Van Dam et al. found that the degree of anxiety and depression of family members with sufficient information and confidence in patient care was significantly lower compared to caregivers with insufficient information and low confidence in patient care. When using CES-D to investigate the family members of cancer patients, it is found that the deterioration of patients' condition, depression, lack of daily action, tension and pain, and high need for care can all lead to family members' depression [29]. Van et al. in a cohort study of 237 family members using CES-D, they believe that young family caregivers have a higher degree of depression. Different stages of diagnosis, surgery, and treatment for patients and different family circumstances will have different family burdens, such as financial status, working hours of family members, and whether there are young children to care for at home. Different family burdens also have different effects on family members' anxiety and depression. Davies et al. POMS Depression scale and anxiety scale were employed to evaluate the family members of patients with hematopoietic stem cell transplantation [30]. The degree of depression and anxiety of the family members at the initial stage of hematopoietic stem cell transplantation was even higher compared to the patients and lasted for 12 months.

The article "Study on the Conduction Analysis and Blocking Intervention Scheme of Emotional Disorders between Cancer Patients and Their Families" was retracted in 2023. Reasons: unreliable results or conclusions; concerns about the data; concerns about the results or conclusions; concerns about the peer review.

The mechanism of diagnosis, intervention, and treatment of doctor-patient-affective disorder refers to the process of influencing the psychological activities, personality characteristics, or psychological problems of a certain object step by step under the guidance of psychological theory, so as to make it change toward the expected goal [30]. With the attention to the psychological state of cancer patients, the diagnosis, intervention, and treatment mechanism of doctor-patient-affective disorder has also been recognized and developed, and effective doctor-patient-affective disorder diagnosis, intervention, and treatment mechanism can promote the immune index of the body [31]. Cancer patients will not only have psychological burden but also cause a series of serious consequences to life, marriage, and family because of a series of expenses and adverse reactions caused by treatment, resulting in psychological burden such as anxiety, depression, and fear. Doctor-patient-emotional disorder diagnosis, intervention, and treatment mechanism has gradually become auxiliary treatment for cancer patients and their families. With the reform of the medical model and the improvement of people's spiritual pursuit, pay attention to the mental health of cancer patients and their families, and promote their life treatment, and psychological intervention has become a seemingly unnecessary but indispensable treatment.

The article "Study on the Conduction Analysis and Blocking Intervention Scheme of Emotional Disorders between Cancer Patients and Their Families" was retracted in 2023. Reasons: unreliable results or conclusions; concerns about the data; concerns about the results or conclusions; concerns about the peer review.

According to previous literature, worrying about patient's condition and prognosis, the impact of long-term care on work, heavy care burden, low income and huge financial burden, taking on more obligations and responsibilities, and other reasons can make cancer patients mainly take care of their relatives to produce adverse psychological stress [31]. The gender of relatives, the status of social support, the functional status, and symptoms of patients are the main influencing factors of adverse psychological stress. This study found that family age, family income status, gender, tumor location, course of disease, TNM stage, and somatic symptoms of patients were the main factors causing anxiety and depression in relatives of cancer patients, which was consistent with the results of previous studies [32]. Liu Aiqin et al. found that the depression and anxiety of relatives of hospitalized cancer patients with poor family financial condition were more serious than those with good economic condition. Studies by Chen Jianhua et al. have also confirmed that economic burden is the most important sign of anxiety and depression in relatives of cancer patients, due to the lack of exact and effective methods for tumor treatment, and it is usually a combination of surgery, chemotherapy, radiotherapy, and other treatment methods, which is expensive. At present, the coverage of medical insurance in our country is narrow, and most of the expenses need to be borne by individuals, which undoubtedly causes a heavy economic burden for the poor relatives and becomes another source of stress leading to the bad stress of the relatives. Relatives may have a sense of uselessness due to insufficient financing of medical expenses, and they may also worry that medical expenses will affect the treatment of patients, resulting in a sense of self-responsibility. The patients with advanced cancer were seriously ill, had many symptoms, and their relatives' care burden and psychological pain were all aggravated. They have to spend more energy and spending with health care staff to try their best to alleviate the suffering of patients, resulting in increased impact on work and daily life and increased financial burden, coupled with the sense of uselessness, hopelessness, and loss caused by relatives who are suffering from illness or dying, and there is nothing they can do about it, which often causes relatives to be in a state of anxiety and depression.

The relatives of cancer patients have a serious state of anxiety, especially the spouses of patients, and relatives who report more somatic symptoms are more likely to have anxiety [33]. Medical staff should pay attention to the mental health status of relatives of cancer patients and actively take targeted intervention measures, such as strengthening psychological security and information support to the spouses of cancer patients, so that they can adopt positive coping styles and build confidence in the treatment of patients. Controlling patient's symptoms early decreases patient's pain and the psychological stress it causes, lessening the negative impact on patient's relatives' mental health and ability to help the patient. In view of the emotional disorders of cancer patients and their families in each stage, according to the attribution analysis, the diagnosis, intervention, and treatment methods of doctor-patient-related emotional disorders were provided, and the classified and accurate intervention scheme was formed by comprehensive use of psychological intervention methods, and the scale feedback is continuously optimized to effectively relieve the emotional disorders of patients and their families, so as to maintain the mental health of patients and their families.

The article "Study on the Conduction Analysis and Blocking Intervention Scheme of Emotional Disorders between Cancer Patients and Their Families" was retracted in 2023. Reasons: unreliable results or conclusions; concerns about the data; concerns about the results or conclusions; concerns about the peer review.

Conclusively, family income status, tumor location, disease course, TNM stage, and somatic symptoms of patients are the risk factors affecting relatives' anxiety and depression. After establishing the diagnosis, intervention, and treatment mechanism of doctor-patient-affective disorder, the emotional disorder of family members of cancer patients is significantly promoted and the intervention satisfaction is high. The scheme is worth popularizing.

## Figures and Tables

**Figure 1:** Comparison of patient satisfaction between the two groups.

**Table 1:** Factors affecting the incidence of anxiety and depression in relatives [*n*/%].

Factors	*n* = 150	Anxiety and depression occur	*χ* ^2^	*P*
Age of the family member (age)				
≤25	20	6 (28.6)	15.278	<0.01
25-50	105	69 (66.2)		
>50	25	8 (33.3)		
Gender of family members				
Male	88	48 (54.8)	0.053	>0.05
Female	62	35 (56.8)		
Family members' years of education (years)				
≤9	52	27 (51.4)	0.536	>0.05
>9	98	57 (58.0)		
Professional status of family members				
Cadres, staff, intellectuals	52	29 (54.9)	2.359	>0.05
Farmers	44	28 (63.2)		
Workers and others	54	26 (48.7)		
The relationship between family members and patients				
Spouse	67	37 (55.3)	4.463	>0.05
Children	72	44 (60.8)		
Other	11	3 (27.3)		
Household income status				
Good	10	4 (40.0)	144.294	<0.01
Medium	88	40 (45.5)		
Difference	52	40 (76.9)		
Payment method of patients' medical expenses				
At one's own expense	78	42 (54.6)	1.039	>0.05
Rural cooperative medical insurance	28	14 (50.0)		
Medical insurance for urban workers	44	27 (61.3)		
Patient sex				
Male	83	58 (69.5)	15.908	<0.01
Female	67	25 (38.3)		
Age of the patient (age)				
<40	30	14 (47.6)	0.453	>0.05
40-60	85	51 (60.0)		
≥60	35	18 (52.0)		
Tumor location				
Digestive system	92	59 (64.6)	10.632	<0.01
Reproductive system	25	7 (27.8)		
Other	33	17 (52.2)		
Course of disease of the patient (month)				
<1	69	40 (57.1)	6.623	<0.01
1-6	55	34 (61.5)		
>6	25	8 (32.0)		
TNM staging of patients				
I-II	82	35 (42.7)	6.290	<0.01
III-IV	68	43 (62.2)		
Somatic symptoms of patients (items)				
<3	55	24 (43.6)	8.727	<0.01
≥3	67	47 (70.1)		
Treatment mode of patients				
Surgical treatment	92	57 (61.5)	3.426	>0.05
Radiotherapy and chemotherapy	58	27 (46.3)		
Patient's knowledge of the disease				
I do not know	40	25 (62.5)	1.160	>0.05
Partial knowledge	47	23 (48.9)		
Fully aware of	64	35 (54.7)		

The article "Study on the Conduction Analysis and Blocking Intervention Scheme of Emotional Disorders between Cancer Patients and Their Families" was retracted in 2023. Reasons: unreliable results or conclusions; concerns about the data; concerns about the results or conclusions; concerns about the peer review.

**Table 2:** Logistic regression analysis of influencing factors of anxiety and depression in relatives.

Variable	*b*	S.E	Chi-square value	*P*	OR	95% CI for OR
Family age	0.733	0.431	2.892	0.089	2.081	0.894-4.844
Household income status	0.533	0.103	26.778	0.001	1.704	1.393-2.085
Patient sex	0.452	1.221	0.137	0.711	1.571	0.144-17.204
Tumor location	1.240	0.316	15.398	0.001	3.456	1.860-5.420
Course of disease	1.330	0.543	5.999	0.014	3.781	1.304-10.960
TNM staging of patients	1.221	0.533	5.248	0.022	3.391	1.193-9.638
Somatic symptoms of patients	1.213	0.355	11.675	0.001	3.364	1.677-6.745

**Table 3:** Comparison of social support between the two groups [$\bar{x}\pm \text{s}$, points].

Group	*N*	Objective support	Subjective support	Support utilization	Total score of social support
C group	75	8.12 ± 0.31	23.12 ± 1.22	7.04 ± 0.12	37.69 ± 2.45
R group	75	9.93 ± 0.56	25.39 ± 1.44	8.33 ± 0.66	42.84 ± 0.77
*t*		24.489	10.416	16.653	17.366
*P*		<0.01	<0.01	<0.01	<0.01

**Table 4:** Comparison of depression scores between the two groups [$\bar{x}\pm \text{s}$, points].

Group	*N*	Before intervention	One week after intervention	2 weeks after intervention	3 weeks after intervention	4 weeks after intervention
C group	75	24.18 ± 0.46	22.69 ± 2.33	20.18 ± 1.56	18.29 ± 1.23	16.48 ± 1.44
R group	75	24.19 ± 0.67	20.18 ± 0.55	17.48 ± 0.21	14.24 ± 0.44	10.83 ± 0.42
*t*		0.106	80.089	14.854	26.849	32.620
*P*		>0.05	<0.01	<0.01	<0.01	<0.01

**Table 5:** comparison of anxiety scores between the two groups [$\bar{x}\pm \text{s}$, points].

Group	N	Before intervention	One week after intervention	2 weeks after intervention	3 weeks after intervention	4 weeks after intervention
C group	75	56.38 ± 1.66	53.82 ± 3.31	48.59 ± 2.14	44.18 ± 1.66	40.78 ± 1.56
R group	75	56.82 ± 1.56	45.38 ± 3.12	42.48 ± 2.54	40.15 ± 3.12	36.42 ± 1.22
*t*		1.672	16.068	15.931	9.875	19.066
*P*		>0.05	<0.01	<0.01	<0.01	<0.01

The article "Study on the Conduction Analysis and Blocking Intervention Scheme of Emotional Disorders between Cancer Patients and Their Families" was retracted in 2023. Reasons: unreliable results or conclusions; concerns about the data; concerns about the results or conclusions; concerns about the peer review.

## Data Availability

No data were used to support this study.
